# The Study of Fetal Rat Model of Intra-Amniotic Isoproterenol Injection Induced Heart Dysfunction and Phenotypic Switch of Contractile Proteins

This article has been retracted.

**DOI:** 10.1155/2014/360687

**Published:** 2014-07-20

**Authors:** Yifei Li, Jie Fang, Yimin Hua, Chuan Wang, Dezhi Mu, Kaiyu Zhou

**Affiliations:** ^1^Department of Pediatric Cardiovascular Disease, West China Second University Hospital, Sichuan University, No. 20, 3rd Section, South Renmin Road, Chengdu, Sichuan 610041, China; ^2^West China Stomatology School, Sichuan University, Chengdu, Sichuan 610041, China; ^3^Ministry of Education Key Laboratory of Women and Children's Diseases and Birth Defects, West China Second University Hospital, Sichuan University, Chengdu, Sichuan 610041, China

## Abstract

To establish a reliable isoproterenol induced heart dysfunction fetal rat model and understand the switches of contractile proteins, 45 pregnant rats were divided into 15 mg/kg-once, 15 mg/kg-twice, sham-operated once, sham-operated twice, and control groups. And 18 adult rats were divided into isoproterenol-treated and control groups. H&E staining, Masson staining, and transmission electron microscope were performed. Apoptotic rate assessed by TUNEL analysis and expressions of ANP, BNP, MMP-2, and CTGF of hearts were measured. Intra-amniotic injections of isoproterenol were supplied on E14.5 and E15.5 for fetuses and 7-day continuous intraperitoneal injections were performed for adults. Then echocardiography was performed with M-mode view assessment on E18.5 and 6 weeks later, respectively. Isoproterenol twice treated fetuses exhibited significant changes in histological evaluation, and mitochondrial damages were significantly severe with increased apoptotic rate. ANP and BNP increased and that of MMP-2 increased in isoproterenol twice treated group compared to control group, without CTGF. The isoforms transition of troponin I and myosin heavy chain of fetal heart dysfunction were opposite to adult procedure. The administration of intra-amniotic isoproterenol to fetal rats could induce heart dysfunction and the regulation of contractile proteins of fetuses was different from adult procedure.

## 1. Introduction

During embryonic heart development, most fetal arrhythmias are transient and benign [1]. However, sustained fetal arrhythmias may result in fetal congestive heart failure and hydrops, even death [2–5]. With the rapid development of fetal echocardiography, accurate prenatal diagnosis for some types of fetal arrhythmia and heart dysfunction can be achieved [6] in collaboration with multiple evaluation systems [7–9]. Although fetal heart dysfunction characterizes with similar histopathological features regardless of their origins, but it seems to be a very different pathophysiological procedure in contrast with adult heart failure. Nowadays, transplacental therapies with digoxin, as well as other cardiovascular drugs, have been used as effective therapeutic alternations to fetal cardiac severe events. And some cohort studies have been conducted with impressed results. However, there are only few studies focused on the complex mechanisms of fetal heart failure and pay no attention to the molecular regulation under this specific procedure [4, 5]. However, there is no research providing a reliable model of fetal heart dysfunction, which limits the further researches on this field. So it is important and urgent to establish a kind of fetal heart dysfunction model and understand its pathophysiology.

Troponin I and myosin heavy chain (MHC) are two kinds of molecular motors both in cardiac and skeletal muscles. There are two phenotypic isoforms of troponin I, cardiac troponin I (cTnI), and slow skeleton troponin I (ssTnI), while there are also two isoforms of MHC, *α*-MHC, and *β*-MHC. As it is known, ssTnI and *β*-MHC are fetal isoforms which are mainly expressed in fetal hearts. The cTnI and *α*-MHC become the domain isoforms of mammalian heart after birth. Unfortunately, many pathological conditions represent a return to fetal gene program [10, 11]. In adult heart failure, previous studies confirmed that the expressions of cTnI and *α*-MHC reduced, while the expressions of ssTnI and *β*-MHC increased resulting in worsening cardiac function [12]. So it was important to get an understanding on how the switches of contractile proteins are during embryonic stage.

## 2. Materials and Methods

### 2.1. Animals

45 female pregnant Sprague-Dawley rats (400–450 g) and 18 normal female ten-week adult Sprague-Dawley rats (250–300 g) were purchased from the Experimental Animal Center of the Sichuan University. This study was completed in accordance with the guidelines on the care and use of animals for research purposes by the Institutional Animal Care and Use Committee of Sichuan University and had been approved by Institutional Animal Care and Use Committee of Sichuan University. Rats were housed within individual metabolism cages in an animal facility with a 12-hour dark/light cycle and controlled temperature and humidity. Water and food were administered unrestricted throughout the study.

### 2.2. Establishment of the Fetal and Adult Heart Dysfunction Model

All 45 pregnant Sprague-Dawley rats were divided into five groups, which were 15 mg/kg once (Iso1) group (*n* = 9), 15 mg/kg twice (Iso2) group (*n* = 9), sham-operated once (Sham1) group (*n* = 9), sham-operated twice (Sham2) group (*n* = 9), and control (Con) group (*n* = 9). Heart dysfunction was induced by two intra-amniotic injections of homologous isoproterenol (ISO) (Sigma, St. Louis, MO, USA) with laparotomy on E14.5 and E15.5 or one single injection with laparotomy on E14.5. The dosage of ISO was calculated according to fetal size, and the average weight on E14.5 was about 2.3 g while the average weight on E15.5 was about 2.7 g. At the same time the normal saline was injected in sham groups following the same experimental procedure. All adult rats were divided into 2 groups, which were continuous ISO injection group (adult Iso) (*n* = 9) and nontreatment group (Adult Con) (*n* = 9). A protocol of continuous 7 days of intraperitoneal injections of ISO as a dosage of 30 mg/kg/day was carried out to build adult heart failure [13, 14]. Rats were lightly anesthetized with 10% chloral hydrate (3 mL/kg, i.p.). The abdomens of maternal rats and chests of adult rats were shaved, and rats were placed on a plant apparatus with fixed posture. All the survival fetal rats were examined by IE33, Philips Ultrasound equipped with an 11 mHz linear transducer, while adult rats were scanned by M-Turbo, Sonosite Ultrasound equipped with an 8 mHz linear transducer. Parasternal long-axis and short-axis views of left ventricle were obtained at an imaging depth of 2.0–2.5 cm on E18.5 for fetuses and 6 weeks after intervention they were completed for adults using the imaging software which came with IE33 and M-Turbo, respectively. LVEFs were calculated according to Teichholtz M-model formula [15], and LVFSs were calculated as (LVDD − LVSD)/LVDD × 100%. For fetus, vertebrae were first identified during ultrasound scanning and obtained views of thoracic cavity by rotating the transducer next, after that finally to make the sectional images of fetal hearts. We defined LVEF reduced 30% as heart dysfunction with Con groups. Besides, left ventricular fractional shortening (LVFS), heart rate (HR), left ventricular end-diastolic dimension (LVDD), left ventricular end-systolic dimension (LVSD), and heart weight/tibia length ratio (HW/TL) have also been assessed to evaluate the cardiac function and morphology of fetal and adult rats.

### 2.3. Tissue Preparation

After echocardiography was performed, all the survival rats were anesthetized with 10% chloral hydrate (3 mL/kg, i.p.). Laparotomies were performed with the fetal units removed rapidly, and the hearts of adults were taken with thoracotomy. Hearts from all rats were rapidly harvested and frozen in liquid nitrogen and stored at −80°C for further analysis. Another piece of heart from each rat was fixed in 4% paraformaldehyde and embedded in paraffin. Besides, one more piece of heart was fixed in 2.5% glutaraldehyde for transmission electron microscope analysis.

### 2.4. Histological Assessment

After 24–48 h in 4% paraformaldehyde, the blocks were dehydrated and embedded in paraffin, cut into 4 *μ*m slices, heated overnight in a 60°C incubator, and then dewaxed and stained with H&E and Masson dye. One slice was chosen from each rat and was analyzed under a microscope. Masson staining for the presence of interstitial collagen fiber accumulation was a marker of cardiac fibrosis. The ratio of interstitial fibrosis to the total left ventricular area was calculated from 20 randomly selected microscopic fields in five individual sections per heart using a camera attached to an Leica DM2000 microscope, with images further analyzed by Image-Pro Plus 5.1 (Media Cybernetics, Silver Spring, MD), excluding coronary vessels and perivascular regions.

Apoptosis in cardiac tissue was determined with the DeadEnd Fluorometric TUNEL System (Promega), which catalytically incorporates fluorescein-12-dUTP at DNA strand breaks as previously described [16]. All sections were counterstained with DAPI (Molecular Probes) at a final concentration of 2 *μ*M. Images were viewed with epifluorescence microscopy (Leica TCS SP5) within 24 hours and analyzed with Image-Pro Plus 5.1 Software (Media Cybernetics, Silver Spring, MD).

### 2.5. Transmission Electron Microscope

Tissues were fixed with glutaraldehyde followed by osmium tetroxide. After being washed with PBS, the tissues were dehydrated in alcohol series, embedded in epoxy resin, sectioned at a thickness of 70 nm, and stained with uranyl acetate and lead citrate. The resultant sections were subjected to examination for ultrastructure using a transmission electron microscope (H-7650, Hitachi, Japan).

Mitochondrial damage was assessed using FLAMENG grading system [17]: 0 = normal matrix granules without visible damage; 1 = loss of matrix granules and light clearing of matrix; 2 = moderate clearing of matrix, moderate swelling, and partial fragmentation of cristae; 3 = severe clearing, severe swelling, and loss of cristae; and 4 = amorphous dense granules. Mitochondrial damage was examined at 5 microscopic fields for each tissue section. The average of the mitochondrial damage grading was used as damage index.

### 2.6. Transcription Analysis

#### 2.6.1. RNA Extraction and cDNA Synthesis

Total RNA was extracted from frozen cardiac tissue by TRIzol (Invitrogen, Life technologies, Carlsbad, CA) and subjected to qualitative and quantitative measurements using a spectrophotometer (GeneQuant 100, GE healthcare). 1 ug of total extracted RNA was reverse transcribed to cDNA using PrimeScript RT reagent kit with gDNA eraser (DRR047A, Takara, Dalian, China) according to the manufacturer's instructions.

#### 2.6.2. Real-Time Quantitative Polymerase Chain Reaction (qPCR)

Real-time (RT) PCR was performed with cDNA templates and SsoFast EvaGreen Supermix (Bio-Rad Laboratories, Hercules, CA). Briefly, sequences were amplified using 5 uL reaction mixture, 0.3 uL forward primer (10 pmol/L), 0.3 uL reverse primer (10 pmol/L), 3.4 uL nuclease-free H_2_O, and 1 uL cDNA in a total volume of 10 uL. PCR conditions were 39 cycles of 30 sec at 95°C, 30 sec at 60°C, and 1 min at 72°C, preceded by an initial denaturation of 3 min at 95°C, and followed by a continuous melt curve from 65–95°C. All the primer sets were tested to ensure the efficiency of amplification over a range of template concentrations. All samples were amplified in triplicate. Expression level of atrial natriuretic peptide (ANP), brain natriuretic peptide (BNP), matrix metalloproteinase- (MMP-) 2, and connective tissue growth factor (CTGF) transcript was represented by the mean of triple tests. The relative expressions of above mRNA were normalized to expression of GAPDH using 2^−ΔΔCt^ method.

The primer sequences used were as follows:

 5′-GGGCTCCTTCTCCATCACC-3′ (ANP-F),
 5′-CTCCAATCCTGTCAATCCTACC-3′ (ANP-R),
 5′-TGGGAAGTCCTAGCCAGTCTC-3′ (BNP-F),
 5′-GCAGCTTGAACTATGTGCCAT-3′ (BNP-R),
 5′-TTACACACCTGACCTGGACCCT-3′ (MMP-2-F),
 5′-CGTTCCCATACTTACTCGGACC-3′ (MMP-2-R),
 5′-CCGGATCCGAGCTTTCTGGCTGCACC-3′ (CTGF-F),
 5′-GGCTGCAGTCTCCGTACATCTTCCTG-3′ (CTGF-R),
 5′-TGAAGTTTTCTGGAGGCGGAG-3′ (cTnI-F),
 5′-TCTCTACCTCTGGAGATCAGCATGG-3′ (cTnI-R),
 5′-AAGCACCTCTACTGCAAGGTTGGG-3′ (ssTnI-F),
 5′-TGCCTCCACAACACGAGAGAGATC-3′ (ssTnI-R),
 5′-ACAGAGTGCTTCGTGCCTGAT-3′ (*α*-MHC-F),
 5′-CGAATTTCGGAGGGTTCTGC-3′ (*α*-MHC-R),
 5′-GCTACCCAACCCTAAGGATGC-3′ (*β*-MHC-F),
 5′-TCTGCCTAAGGTGCTGTTTCA-3′ (*β*-MHC-R),
 5′-CAGGGTCGACCTTGCCCACAGCCTT-3′ (GAPDH-F),
 5′-GCCAAGGATATCCATGACAACT-3′ (GAPDH-R).

### 2.7. Western Blot Analysis

50 mg tissues of pooled 5-6 fetal hearts and 100 mg tissues from an adult heart were homogenized in buffer containing 0.3 mL and 1 mL RIPA, respectively, (P0013B, Beyotime) with 1% complete protease inhibitor cocktail (P8340, Sigma-Aldrich). The homogenate was then centrifuged at 12,000 g for 5 min at 4°C. Protein concentration was determined using enhanced BCA protein assay kit (P0010S, Beyotime) according to the manufacturer's protocol. Total protein (25 *μ*g/lane) was separated on 8% SDS-polyacrylamide gel and transferred to polyvinylidene fluoride (PVDF) membranes (ISEQ00010, Millipore). The membranes were blocked in 5% BSA in phosphate-buffered saline containing 0.1% Tween-20 (PBST). Thereafter, blocked membranes were incubated overnight at 4°C with monoclonal primary antibody for cTnI (sc-31655, Santa Cruz Biotechnology, 1 : 200), ssTnI (sc-8119, Santa Cruz Biotechnology, 1 : 200), *α*-MHC (sc-168676, Santa Cruz Biotechnology, 1 : 200), *β*-MHC (sc-168678, Santa Cruz Biotechnology, 1 : 200), and GAPDH (ab8245, Abcam, 1 : 7500). Following extensive washing with PBST, membranes were incubated with a 1 : 10000 dilution of donkey anti-goat IgG secondary antibody and goat anti-mouse IgG secondary antibody (sc-2020, Santa Cruz Biotechnology and ZB-2305, ZSGB-BIO). After extensive washing with PBST, protein-antibody complexes were visualized by ECL method.

### 2.8. Statistical Analysis

The SPSS program software (version 20.0, SPSS Inc.) was used for statistical analysis. Quantitative data were expressed as mean ± SEM. One-way ANOVA was used to analyze the difference among groups. The difference among each group was analyzed with* U* test with Bonferroni correction. The difference was considered significant when *P* < 0.05.

## 3. Results

### 3.1. Clinical Findings

All pregnant female rats developed well, and no one died according to surgery performed. However, one rat of Iso1 group and 2 rats from Iso2 group suffered premature delivery. And 7 fetuses in Iso2 group died inside of the uterus, while 3 fetuses in Iso1 group and 3 fetuses in Sham1 group died. There was no dead case in Sham2 and Con groups. As there were usually more than 10 fetuses in a maternal rat, it was available to collect 9 samples for all the groups in each analysis even there were 2 maternal rats that suffered premature delivery. During the duration of the study, 3 maternal animals lost weight and exhibited signs of chronic dehydration. During the establishment of adult heart failure, only 1 case died (11.1%, 1/9) in adult Iso group, while all rats were alive in Con group. Meanwhile, the assessment of HW/TL had been carried out to evaluate the hypertrophy of adult failing heats. Results showed that the failing adult hearts developed with a significantly increased HW/TL (Table 1).

### 3.2. Echocardiography

The structure of cardiac chambers and aorta are shown in Figures 1(a) and 1(b). Representative M-mode echocardiographic image from fetal animal on E18.5 after initiating ISO is shown in Figures 1(e)–1(h). Worsening of LVEFs was observed in Iso2 groups. These data were all collected under chloral hydrate anesthesia. In the subset of fetus that achieved target LVEF, there was significant exacerbation of all echocardiographic parameters of ISO injection (Table 1). Mild LV hypertrophy was observed along with a much more profound reduction in systolic and diastolic contraction and shortening fraction. Besides, worsening of LVEFs was observed in animals of adult Iso group (Figures 1(c) and 1(d) and Table 1). Moreover, the worsening LVFS, LVDD, and LVSD demonstrated that there were damages of diastolic function among ISO-treated fetal and adult rats (Table 1).

### 3.3. Histological Assessment

On the day of E18.5, the interstitial fibrosis rates were, respectively, 13.0 ± 0.9% in Iso1 group, 21.7 ± 2.6% in Iso2 group, 12.3 ± 1.2% in Sham1 group, 11.3 ± 1.8% in Sham2 group, and 10.6 ± 1.4% in Con group (Figures 2(a) and 2(b)). We also measured the morphology of cardiomyocytes and myocardium of whole ventricular area among five experimental groups using H&E staining (Figure 3). In ISO-treated hearts, cardiomyocytes were hypertrophic and nonuniform in shape with disorganized arrangement. In control hearts, cardiomyocytes were of a uniform size and shape, and interstitial space was clearly visible as dark, variegated bands throughout the myocardium.  Figure 4(a) demonstrates representative TUNEL stains from control to ISO-treated hearts and the overall apoptotic cells number per microscopic field in any area of fetal heart as they were quite a small tissue. As compared to control group, ISO treatment enhanced cardiomyocytes apoptosis in hearts (apoptotic cells number per microscopic field of Iso1, Iso2, Sham1, Sham2, and Con was 21.63 ± 1.27, 30.10 ± 3.11, 9.30 ± 3.01, 5.30 ± 0.95, and 5.51 ± 0.76, respectively; Figure 4(b)). This increase was statistically significant in the Iso2 group (*P* < 0.0001).

### 3.4. Transmission Electron Microscope and Damage Evaluation

To further evaluate the impacts of ISO induced cardiac dysfunction on heart microstructure, we examined the ultrastructure of the heart using a transmission electron microscope of fetuses among five groups on E18.5 (Figure 5(a)). The myocardial damages were analyzed based on the myocardial and mitochondria morphological changes (FLAMENG index of Iso1, Iso2, Sham1, Sham2, and Con were 1.28 ± 0.07, 3.05 ± 0.09, 0.61 ± 0.08, 0.91 ± 0.11, and 0.63 ± 0.12, respectively; Figure 5(b)). As shown in Figure 5(a), myocardial vacuolization, degranulation of endoplasmic reticulum, and mitochondrial damages were observed in the fetal hearts of ISO injected groups with a varied extent. Specifically, severe reshaping, severe swelling, and loss of cristae with amorphous dense granules were observed in Iso2 group indicating severe mitochondrial damages. Statistical comparisons revealed that significant differences existed between fetuses with ISO injection and fetuses with sham-operated as well as normal fetuses. However, no difference was recorded on fetuses among sham groups and normal group.

### 3.5. Transcriptional Expression of Heart Failure Biomarkers

In contrast to what is previously discussed, ISO-treated hearts did not exhibit clear cardiomyocyte borders, and interstitial connective tissue volume was markedly diminished. To explore this further, we examined myocardial gene expression of CTGF and MMP-2, which would be expected to augment collagen degradation (Figures 6(a) and 6(b)). As compared with control hearts, CTGF expression was unchanged in ISO-treated hearts, whereas MMP-2 expression was significantly (*P* < 0.05) upregulated. The rapid increase of MMP-2 would be expected to favor collagen turnover and loss, which was consistent with the histological findings in Figure 3.

Moreover, the mRNA expression of ANP and BNP was recorded to confirm that this was an exact model of fetal heart dysfunction (Figures 6(c) and 6(d)). The increase of BNP was statistically significant (*P* < 0.01) in Iso2 groups but not statistically significant in Iso1 group. That could give more efficient evidence on fetal heart dysfunction of intra-amniotic ISO injection. Consistent with these histological findings of hypertrophy, mRNA expression of ANP, a hypertrophic marker, was increased by 2.5-fold in ISO-treated hearts as compared with control.

### 3.6. Expression of Contractile Proteins between Fetal and Adult Heart Failure

Interestingly, in fetal Iso2 group, ssTnI was repressed compared to normal fetal rats (*P* < 0.01), while *α*-MHC was increased according to western blot analysis, while there was no change in cTnI and *β*-MHC expressions. Besides, the elevated ratios of cTnI/ssTnI and *α*-MHC/*β*-MHC level were identified (*P* < 0.01) (Figure 7). And the same evaluating procedures were performed in adult ones. As same as previous studies, we found that the level of cTnI and *α*-MHC dropped in adult Iso rats (*P* < 0.01), while elevating level of ssTnI and *β*-MHC had been confirmed (*P* < 0.01) with decreasing ratio of cTnI/ssTnI and *α*-MHC/*β*-MHC (*P* < 0.01) (Figure 7). Besides, RT-PCR was enrolled for mRNA analysis for cTnI, ssTnI, *α*-MHC, and *β*-MHC, which had the results consistent with western blot analysis (Figure 8).

## 4. Discussion

In this study, we reported a stable model of ISO induced fetal heart dysfunction in rats for the very first time. Specifically, consecutive two intra-amniotic injections of ISO induced (1) an impaired LV contraction and relaxation, (2) hypertrophic, reshaping, and disorganized cardiomyocytes, (3) increased interstitial fibrosis, (4) increased cardiac cell apoptotic rate, (5) severe mitochondrial damages, and (6) elevated expressions of MMP-2, ANP, and BNP. All the assessed features were hallmarks of a failing heart. The ISO induced adult heart failure model was generally used to analysis pathophysiological changes. So the establishment of fetal heart dysfunction model might be used as a platform to explore acute, chronic, and even postnatal pathophysiologic responses to abnormal hemodynamics in the context of fetal heart dysfunction.

To build a reliable model of adult heart failure many protocols had been reported, including coronary artery ligation, abdominal aorta coarctation, and doxorubicin-induced and large dose ISO administration [18–21]. In contrast with adult heart dysfunction which was primarily caused by myocardial infarction, hypertension and cardiomyopathy, the fetal heart dysfunction is mainly caused by abnormal hemodynamics and arrhythmias. Limited by the specific condition of fetuses, it was impossible to achieve coronary artery ligation and abdominal aorta coarctation by surgery even under microscope. However, doxorubicin was proven as a kind of cytotoxicity medication, and the administration of doxorubicin would result in severe interferences to fetal development, which might lead to much more severe injuries far beyond hearts itself. The administration of ISO, a *β*-adrenergic receptor agonist, induces cardiac remodeling with left ventricular hypertrophy and fibrosis. It was considered as a reliable and acceptable method to establish heart dysfunction model for exploring secrets even with no obvious advantage and disadvantage [13, 14, 22, 23]. In this study we compared the results of two different injection methods to induce fetal heart dysfunction and cardiac remodeling in fetal rats. Moreover, we found that only 2-3 days which was quite less than the waiting time to build an adult model were available to make cardiac dysfunction and myocardial remodeling after intra-amniotic ISO injections with great increase of ANP and BNP which were highly specific biomarkers of heart dysfunction [24]. We considered that it was fetuses that were more sensitive to the changes around and the hearts were going on their developmental procedure, so that the remodeling could occur in a limited time. Although heart failure was not identified in Iso1 group, some mild damages such as increased apoptosis rate and FLAMENG index were observed. The results suggested that ISO-treated once could result in some injuries to cardiomyocytes, which was not sufficient to establish a heart failure. This method of ISO induced heart failure might be dose and time dependent. According to previous studies, it was difficult for ISO to cross placenta barrier with a quite low transfer rate. It was impossible to get the fetuses exposed to high concentration of ISO via maternal ISO administration [25, 26]. So we chose intra-amniotic fluid injection to ensure that fetus could receive enough concentration of ISO and a low concentration in maternal circulation. Moreover, we also performed the echocardiography to evaluate maternal cardiac function and confirmed that there were no functional impacts.

In addition, large dose ISO could induce the similar myocardial damage with acute myocardial infarction (AMI) in adult rat heart resulting in heart muscle necrosis and elevated serum troponin. The large dose ISO model was therefore used as a noninvasive AMI model. This suggested that large dose ISO induced heart failure rat model could also be used as heart failure model induced by AMI [27]. Furthermore, previous study found that the elevated expressions of osteoprotegerin (OPG) and receptor activator of nuclear factor-*κ*B ligand (RANKL) in experimental autoimmune myocarditis (EAM) induced heart dysfunction rat model, and anti-IL-17 treatment could change the expressions of OPG and RANKL in ISO induced adult heart dysfunction rat model [28, 29]. And also, ISO injection led the increase of cardiac load. Above description suggested that large dose ISO induced heart dysfunction rat model might share some similar pathophysiological characters with myocardium ischemia, EAM, and overload induced heart failure. Arrhythmias of fetus especially tachyarrhythmia, which could result in myocardium ischemia [7, 30, 31]. Besides, congenital heart disease as well as severe thalassemia could cause harmful hemodynamics which increased cardiac load [32–35]. So it was suggested that large dose ISO induced fetal heart dysfunctional rat model could also share some similar pathophysiological characters with clinical human fetal heart dysfunctional procedure. Therefore, this kind of consideration would support the catholicity and practicability of this firstly fetal heart dysfunctional rat model.

Myocardial apoptosis and mitochondria damages both contribute to myocardial dysfunction in anthracycline and doxorubicin induced heart dysfunction [36–38]. Indeed, ISO-treated fetal rat hearts in our study exhibited both a 5- to 6-fold increase in apoptotic rate and significant increase in mitochondria damage index as quantified by regional microsphere distribution. As prior work demonstrated that doxorubicin can induce apoptosis of cardiomyocytes and result in heart dysfunction, this was also recorded in our model. As myopathic hearts generally showed augmented interstitial fibrosis, prior work demonstrated that MMP in the heart was elevated in a failing heart. Indeed, in this study, the expression of CTGF was unchanged, whereas MMP-2 (which promotes collagen breakdown) was induced, consistent with prior observations. Hence, the interstitial remodeling after ISO exposure was depending on the stage of progression of ventricular remodeling. In adult heart dysfunction model, the longer the period after ISO supplementation is, the more augmented collagen deposition and greater fibrosis formation could be observed. However, our results might describe the greatest remodeled structure for a fetal model during limited pregnant days with some fibrosis formation, which was still much less than adult procedure. The expression of CTGF was related to interstitial fibrosis formation. However, in our study we did not confirm this relationship in fetal model. It might be different between fetal and adult heart remodeling. Nowadays histone deacetylases were proved to be involved in interstitial fibrosis formation [39, 40], and other factors had also been identified [41], so it was considered that the fibrosis in fetal hearts was generated by other pathways.

The contractile velocity of cardiac muscle correlated with composition of troponin and MHC isoforms, suggesting a causal relationship between troponin isoform composition and cardiac contractility. And once the composition of isoforms changed, the heart might result in dysfunction and pathological procedure. Transitions in cardiac contractile isoforms had been identified in response to various adult pathological and physiologic stimuli. Many of these stimuli resulted in cardiac hypertrophy and heart failure accompanying with several changes in gene expression and morphology of cardiomyocytes. Previous studies strongly confirmed that ssTnI and *β*-MHC could be reactivated in adult pathological procedure, which were inactivated in normal adult heart since heart development completed [12, 42]. In our study, we attempted to obtain an essential understanding about the molecular switches under fetal heart failure, especially the differences between fetal and adult procedures. To our great surprise, ssTnI was recorded repression and *α*-MHC was strongly activated during fetal heart failure which was quite different from the knowledge recorded during adult heart failure. However, the expressions of cTnI and *β*-MHC kept stable during fetal heart failure which were still different from adult procedure which showed significant changes. Antithetical transition of the ratio of cTnI/ssTnI and *α*-MHC/*β*-MHC were recorded between fetal and adult heart failure. Kim et al. [43] reported that cTnI could be undetected in adult failing heart. Du et al. [44] confirmed this result in their research. Moreover, Lowes et al. [45] reported that *α*-MHC dropped in adult failing heart consistent with the report from Miyata et al. [46]. The transition of the ratio of cTnI/ssTnI and *α*-MHC/*β*-MHC in adult failing hearts which showed a return to “fetal gene program” was a kind of symbol of adult heart pathology. However, our amazing result recorded an opposite regulation of cTnI/ssTnI and *α*-MHC/*β*-MHC in fetal failing heart to adult ones suggesting a different gene program activated. As the expressions of contractile proteins might be different between human and rat, our results should be limited to rat hearts, and such researches on human were urgently needed.

Huang et al. [47] reported that cTnI null mice could survive longer beyond postnatal day 14 only with ssTnI expression. So it was suggested that the transition of isoforms of troponin I was very important in development and to maintain their life. It was unknown whether fetuses could benefit from such regulation of contractile proteins or not. According to previous studies many transcript factors such as YY-1, Hand1/2, and Smad made some contribution to the regulation of contractile gene expression during adult heart failure [48, 49]. Moreover YY-1 could play different roles in several stages [50]. So such mechanisms might be involved in antithetical regulation of ssTnI and *α*-MHC. And there need a further exploration to find the answer.

There were still some limitations which were as follows: the maternal rats might face the risk of premature pregnancy, without survival neonates after ISO injection. So the information of heart dysfunctional neonates was lacking. And it was impossible to weigh the fetuses inside of the uterus; the weight of fetuses which were used for dosage calculation was converted by embryonic days and the length of body. As twice laparotomy performed within Iso2 and Sham2 groups, there might be some free gas between skin and subcutaneous tissue. So it was impossible to get echocardiographic images as clear as Con group under Philips IE33 ultrasound system.

## 5. Conclusion

We concluded that administration of intra-amniotic ISO twice as a dosage of 15 mg/kg to fetal rats induced heart dysfunction. And these ISO twice treated fetuses exhibited significant dysfunction by fetal echocardiography with significant changes in histological evaluation and the expressions of multiple heart failing and remodeling genes. This clinically relevant model was available for exploring pathophysiological responses during fetal heart dysfunction. Moreover, we found that the pathophysiological procedure of fetus was quite different from adult procedure. SsTnI was repressed and *α*-MHC was elevated during fetal heart dysfunction while opposite regulation should be observed during adult procedure. However, its impacts on cardiac function and their postnatal life were still unknown calling for further investigations.

## Figures and Tables

**Figure 1:** Hemodynamic measurements on experimental animals with ultrasound. The structure of cardiac chambers and aorta were shown in (a) and (b); representative M-mode echocardiographic image from fetal heart on E18.5 was shown in C-H along with M-mode echocardiographic image from adult heart 6 weeks after ISO injection. (c) For adult Iso, (d) for adult Con, (e) for Iso1, (f) for Iso2, (g) for Sham2, and (h) for Con. The image of Sham1 was not presented with limited space. LV, left ventricle; RV, right ventricle.

**Figure 2:** The comparison of myocardial fibrosis rate in all experimental groups: (a), Masson stain, and interstitial fibrosis occurred obviously in Iso2 group, ×400; (b), interstitial fibrosis rate across five groups, the Iso2 group demonstrated a significant higher rate compared to others. ∗*P* < 0.05, ∗∗*P* < 0.01, ∗∗∗*P* < 0.0001. *n* = 4/group.

**Figure 3:** The comparison of morphology in all experimental groups; H&E staining showed that, in ISO-treated hearts, myocytes were hypertrophic and nonuniform in shape with disorganized myocardium myocytes. In control hearts, myocytes were of a uniform size and shape, and interstitial space was clearly visible as dark, variegated bands throughout the myocardium, ×400.

**Figure 4:** Myocardial apoptotic cell number determined with TUNEL staining in control, sham-operated, and ISO-treated hearts. (a) Presented TUNEL staining (with DAPI costaining) in control and ISO-treated hearts. Nuclei are stained blue. TUNEL positive nuclei are green/cyan ×200. (b) Demonstrated apoptotic cell number per microscopic field. ∗*P* < 0.05, ∗∗*P* < 0.01, ∗∗∗*P* < 0.0001. *n* = 4/group.

**Figure 5:** Mitochondrial damages determined with transmission electron microscope in control, sham-operated, and ISO-treated hearts. (a) Presented transmission electron microscope images in control and ISO-treated hearts. Areas of mitochondria were focused. Severe reshaping, severe swelling, and loss of cristae with amorphous dense granules were observed in Iso2 group. 16000x–20000x. (b) Demonstrated FLAMENG index among five experimental groups. ∗*P* < 0.05, ∗∗*P* < 0.01, ∗∗∗*P* < 0.0001. *n* = 3/group.

**Figure 6:** mRNA expression of CTGF, MMP-2, ANP, and BNP in control sham-operated and ISO-treated hearts as quantified by real-time PCR. Individual gene expression was normalized to GAPDH mRNA and displayed as a percentage of control. ∗*P* < 0.05, ∗∗*P* < 0.01, ∗∗∗*P* < 0.0001. *n* = 9/group.

**Figure 7:** Western blot of cTnI, ssTnI, *α*-MHC, and *β*-MHC expression in fetal Iso2, fetal Con, adult Iso, and adult Con hearts. Individual protein expression was normalized to GAPDH expression and displayed as a percentage of control. ∗*P* < 0.05, ∗∗*P* < 0.01, ∗∗∗*P* < 0.0001. *n* = 9/group, while *n* = 8 for adult Iso group.

**Figure 8:** mRNA expressions of cTnI, ssTnI, *α*-MHC, and *β*-MHC expression in fetal Iso2, fetal Con, adult Iso, and adult Con hearts as quantified by real-time PCR. (a) For troponin I of fetuses, (b) for MHC of fetuses, (c) for troponin I of adults, and (d) for MHC of adults. Individual gene expression was normalized to GAPDH mRNA and displayed as a percent of control. ∗*P* < 0.05, ∗∗*P* < 0.01, ∗∗∗*P* < 0.0001. *n* = 9/group, while *n* = 8 for adult Iso group.

**Table 1:** Echocardiography parameters in fetal and adult rats.

	Iso1	Iso2	Sham1	Sham2	Con	Adult Iso	Adult Con
LVEF (%)	89.3 ± 1.5	62.2 ± 5.6***	90.2 ± 1.6	89.9 ± 1.0	89.7 ± 2.6	65.9 ± 2.6***	91.3 ± 2.3
LVFS (%)	52.4 ± 2.1	27.9 ± 3.4**	53.9 ± 2.4	53.1 ± 1.5	54.4 ± 4.1	29.1 ± 1.6*	54.3 ± 2.6
HR	209.2 ± 7.6	247.3 ± 6.3***	204.3 ± 4.4	208.7 ± 8.4	198.7 ± 6.3	206.1 ± 10.1**	159.2 ± 8.8
LVDD (mm)	1.69 ± 0.03	2.15 ± 0.08**	1.70 ± 0.10	1.74 ± 0.07	1.77 ± 0.11	6.40 ± 0.11*	5.94 ± 0.12
LVSD (mm)	0.81 ± 0.04	1.54 ± 0.05***	0.78 ± 0.03	0.82 ± 0.04	0.79 ± 0.05	4.54 ± 0.08***	2.71 ± 0.05
HW/TL (mg/cm)	—	—	—	—	—	166.13 ± 3.86***	75.53 ± 5.51

Achieved echocardiography parameters of fetal and adult rat hearts. Worsening of indicators was observed in Iso2 and adult Iso group compared to normal ones. *P < 0.05, **P < 0.01, and ***P < 0.0001 indicated that there were significant differences between such group and control group. LVEF, left ventricular ejection fraction; LVFS, left ventricular fractional shortening; LVDD, left ventricular end-diastolic dimension; LVSD, left ventricular end-systolic dimension; HW/TL, heart weight/tibia length ratio.
